# Construction Path of Academic English Learning Environment in Colleges and Universities from the Perspective of Education Ecology

**DOI:** 10.1155/2022/6727334

**Published:** 2022-08-25

**Authors:** Jie Hua

**Affiliations:** Faculty of Foreign Languages, Huaiyin Institute of Technology, Huai'an, Jiangsu 223001, China

## Abstract

This paper probes into the construction of academic English learning environment in colleges and universities from the perspective of educational ecology. This paper aims to construct academic English learning environment from the perspective of educational ecology by constructing a teaching community, organizing learning activities, using tool mediation, and optimizing the social and material environment. Understand the construction effect through a questionnaire survey. The results show that among the 1000 surveyed students' average satisfaction with the five elements of the learning environment, the teaching community is 4.6355, the learning community is 4.8963, the learning activity is 4.6987, the tool intermediary is 4.9258, and the social material environment is 4.2536, indicating that the students' satisfaction is high. From the perspective of educational ecology, the construction of academic English learning environment in colleges and universities can effectively optimize teaching and learning community and help to enhance students' motivation, cultivate learning interest, and improve practical ability. The construction effect is worthy of recognition.

## 1. Introduction

Establishing a good academic ecological environment in colleges and universities is conducive to promoting the sustainable development of colleges and universities as a whole. Therefore, relevant managers need to strengthen the construction of academic ecological environment in colleges and universities, clarify the importance and practical significance of establishing academic ecological environment in colleges and universities, and strengthen the handling of various details, so as to build a free, open and standardized academic ecological environment in colleges and universities, and promote the improvement of academic level in colleges and universities. The construction of academic ecological environment in colleges and universities can not only scientifically allocate academic resources to colleges and universities but also achieve the goal of cultivating innovative talents and meet the requirements of education in colleges and universities. Therefore, in the current era, it is very important to carry out the construction of academic ecological environment in colleges and universities [1, 2]. Relevant administrators need to clarify their own management responsibilities, start with the problems of the construction of academic ecological environment in traditional colleges and universities, put forward targeted solutions, and strengthen the research on the construction of academic ecological environment.  Figure 1 shows the proportion of people engaged in academic research in different industries.

During the construction of academic ecological environment in colleges and universities, relevant managers need to clarify the meaning of academic ecological environment construction so as to ensure the orderly progress of follow-up work. First of all, the construction of a harmonious academic ecological environment is mainly to establish a fair competition, democratic, and free academic environment within the scope of the university so that every student and teacher can improve their creative ability according to their own professional ability and knowledge base, which not only is conducive to the realization of personal development but also improves the quality of running a university as a whole. Secondly, relevant managers should formulate innovation reward policies to reward innovative academic research results so that every student and teacher can improve their innovation ability in the school and improve the quality of talent training in colleges and universities. Finally, relevant managers should also create a harmonious interpersonal academic environment within the scope of the university. By cultivating academic teams and research groups, students are encouraged to explore and study academic knowledge, which will help to promote the improvement of the academic level of the university and promote the long-term development of the university [3, 4].

## 2. Literature Review

For a long time, public English teaching for postgraduates has followed the college general English teaching curriculum system, which is divorced from the needs of society and postgraduates for English and has not formed a curriculum system for the characteristics and training objectives of postgraduates, which cannot meet the requirements of cultivating postgraduates' diversified communicative competence, resulting in a great waste of class hours and teaching resources.  Figure 2 shows the sharing mode of teaching resources.

In order to improve the above problems, many scholars have proposed that foreign language teaching for postgraduates should focus on cultivating students' academic communication ability and application ability of professional language, that is, the ability to skillfully acquire and exchange professional knowledge and information by using a foreign language as a tool. Therefore, the construction of an academic English curriculum has become the focus of Public English Teaching Reform for postgraduates. In order to build a teaching staff of academic English and ensure the teaching quality, many colleges and universities have carried out cooperative teaching of academic English between foreign language teachers, subject teachers, and foreign teachers. However, in the existing graduate academic English curriculum system, although Chinese and foreign teachers, subject teachers, and foreign language teachers cooperate in teaching, the content and design are independent and lack connection, and the whole curriculum system is cumbersome and complex [5].  Figure 3 shows the proportion of male and female English teachers.

As academic newcomers and foreign language users, postgraduates face pressure and challenges from both academic and linguistic aspects, and their learning environment is significantly different from that of undergraduates. With the change of tutor responsibility system and teaching objectives, learning is no longer limited to the classroom environment, but a process of meaning construction by learners in the environment of multiple resource systems and multiple forms. The subject to be studied is how to integrate teaching resources more effectively, give full play to the advantages and specialties of teachers, establish the relationship between teaching resources, teacher resources, and learners, and enable learners to obtain the maximum learning benefits. Compared with the curriculum, the design and construction of learning environment plays a more important role in graduate students' foreign language learning and discipline cultivation. Learning environment is “a place where learners use a variety of tools, information, and resources to work together and support each other in order to achieve learning objectives and problem-solving activities.” Behaviorist learning view emphasizes the stimulating effect of environment on learners. Once the external environment stimulation stops, learning behavior will also fade. Behaviorism learning environment mainly aims at the memory, repetition, and behavior acquisition of knowledge concepts. The cognitive learning view holds that learning is a complex information processing process within learners [6, 7]. It is an active psychological process to obtain the symbolic representation of the external environment through the change of brain cognition. The design of learning environment under the cognitive learning view emphasizes that students study and think meaningfully and independently in the environment. Constructivist learning theory holds that “individual” is the main body of construction and “environment” is only the condition and support in the process of individual construction. The two are independent, and their focus is still on individual construction. Therefore, no matter behaviorism, cognitivism, or constructivism, they all emphasize people-centered learning but ignore the integration and common development of human and environment. However, in the view of educational ecological learning, the learning subject has also become an element of the learning environment. The learning environment is an ecological learning system composed of learners, learning activities, tool intermediary system, and social and material environment. The behavior interaction and relationship interaction between various elements are a dynamic cultural ecological environment. The learning environment under the theory of educational ecology puts more emphasis on resource sharing and meaning sharing between subjects and between subject environments and attaches importance to the dynamic correlation and common development between people and various elements of the environment [8–10].  Figure 4 shows the general teaching process.

The “affinities” in the theory of educational ecology was created by the ecological psychologist Gibson. It is defined as all the positive or negative relationships that the environment gives, provides, and configures for the organisms in it. The ecological concept holds that the environment provides resources and opportunities for the actions of organic life, and organisms perceive information content from the environment to guide their actions. In the field of foreign language learning, van Lier pointed out that provision is the opportunities, resources, and support that people can get in the environment in the process of learning action. It is also the interactive learning opportunities and resources that teachers provide in different environments. To sum up, provision is all the material content that language learners can transform the matched potential learning resources and interactive learning opportunities into meaningful positive or negative language learning through behavior in the environment. Therefore, the design of the learning environment needs to consider the learners' own abilities and needs and provide resources, opportunities, and support that match their learning effectiveness, perception, experience, and cognition so that they can obtain meaningful and positive supplies and form a virtuous circle of learning ecology [11].  Figure 5 shows the composition of learning effectiveness.

Based on the learning environment elements and provision theory of the educational ecological learning view, this study takes the training of international and research-oriented talents as the goal, focuses on the international academic exchange ability, and redesigns the learning environment of international academic exchange English, so that all teachers and learners can become factors in the learning environment, interact with each other, and provide students with matching learning opportunities, interaction, and support from both subject content and language. From the perspective of educational ecology, this paper will reconstruct the public foreign language education practice of postgraduates from the four elements of learning environment: teaching community, learning activities, tool intermediary, and social and material environment [12].  Figure 6 shows the teaching process of the Mu class.

## 3. Research Methods

Each teacher and student has a different niche, and different niche has certain advantages. The greater the degree of niche separation, the greater the chance of coexistence. In the past, people paid too much attention to and made use of the overlap and competition between niches, but the really important thing is the coexistence relationship. At present, learning tools such as MOOC and flipped classroom need to be used to effectively connect the classroom and extracurricular so as to provide content support for students' autonomous learning and ubiquitous learning so as to establish a unique cooperative teaching mode chain of graduate academic English. In order to make more efficient use of scarce teachers and implement regional ecological integration development, colleges and universities in Jiangsu Province have also established a teaching cooperation community to share foreign teacher resources, jointly hold competitions, and build a broader external overall learning environment [13, 14].

### 3.1. Teaching Community

The teacher teaching community is a joint organization jointly built by full-time English teachers (main teachers, hereinafter referred to as “Chinese teachers”), subject teachers, foreign teachers (native speakers of English, hereinafter referred to as “foreign teachers”), and teaching assistants, aiming to promote teachers' effective teaching and professional growth through dialogue, cooperation, and sharing activities. Under the theory of educational ecology and the framework of “one body and two wings,” each teacher has a different niche in the whole teaching environment, has different roles, and cooperates and interacts with each other in teaching. As the main body of the implementation of the “one body, two wings” middle school curriculum, Chinese teachers need to always maintain cooperation and dialogue with foreign teachers and subject teachers in a series of links from the demand investigation, planning, formulation, and implementation process to test summary of the academic English curriculum. As one of the “two wings,” subject teachers need to drive, lead, and improve the ability of graduate students to communicate in English. In addition to providing the professional needs of graduate students, it will also guide and encourage students' international academic exchanges in the form of lectures and seminars, taking their own research process as an example. As the other wing of the “two wings,” foreign teachers maintain dialogue and discussion with Chinese teachers and subject teachers in cross-cultural exchanges, international academic norms, and standardization and carry out targeted teaching in the form of a series of special courses embedded in the whole academic English course. Chinese teachers, foreign teachers, subject teachers, and teaching assistants cooperate and communicate closely in the whole teaching activities [15].

Chinese and foreign teachers listen to each other and prepare and discuss lessons collectively every two weeks. Subject teachers and Chinese teachers establish contact and maintain interaction at the beginning, middle, and end of the period. Subject teachers select classic English papers of the subject as teaching materials, and Chinese teachers integrate the existing teaching materials after analyzing the linguistic characteristics of the genre. The teaching assistants participate in the lesson preparation activities arranged by the Chinese teachers, complete the tasks of listening and teaching, and submit the teaching situation briefing to the Chinese teachers every week. The student learning community is the internal environment of the teaching ecology. The learner is not only the learning subject but also the key element in the learning environment. When the graduate student ontology interacts with other elements in the learning environment, it also constitutes the internal learning environment and carries out its own interaction and cooperation. In addition to the rights and responsibilities of teachers and schools in designing the school environment, learners also need to design their own learning environment and actively seek supplies in the environment in combination with their own learning efficiency. In addition to clarifying the surrounding foreign language learning environment and making full use of communication and learning opportunities, graduate students also set up learning groups to carry out collaborative learning driven by projects and tasks. The principle of grouping is homogeneity between groups and heterogeneity within groups. Each group of students has different niches and undertakes different roles and tasks, but they should try their best to achieve the optimization of the results of the group tasks. Therefore, each group of members cooperates, shares, and inspires each other, providing rich supplies for the group members and improving their language application ability and communication ability. After the task is completed, students will conduct self-evaluation, class mutual evaluation, and group mutual evaluation on the task implementation process, results, and learning effects. Excellent group achievements will be selected, displayed, and demonstrated in school level and municipal level activities to create a benign and mutually beneficial learning atmosphere [16, 17].

### 3.2. Learning Activities

Establishing the connection between teachers' teaching community and students' learning community through learning activities is an important link in the design of ecological learning environment. The learning activities must be authentic, specific, and accessible. In the activities, the language skills necessary for postgraduates to conduct international scientific research, innovation, and entrepreneurship must be trained. In specific learning activities, learners will constantly look for the provisions of the learning environment and take actions. Learning activities need to make learners understand their intentions and take the corresponding incentive and restraint measures to stimulate learners' learning intentions and make their actions meet expectations. Each learning activity forms a corresponding teaching module, which is refined into multiple specific learning tasks.

### 3.3. Tool Intermediary

The activities and organic links between the communities need a lot of interaction, communication, and consultation, so the community is full of vitality and vigor. Tool mediation can achieve better quality and effective circulation and connection in the community connection of learning environment [18]. Therefore, in addition to taking the classroom as a basic tool and intermediary system, we have also designed WeChat public platform, MOOC, and other digital information tools to build an ecological learning environment, aiming to facilitate the dynamic, distributed, and efficient connection and interaction between various elements of the learning environment. Among all kinds of tools, it is also important to use the calculation formula. Taking the corpus in English learning as an example, the formula is as follows:

(1) $$\begin{array}{c} C=\left\{s1,s2\ldots ,Sn\right\}. \end{array}$$

In the above formula, C represents the corpus, *s* represents the sentences, and *i* represents the number of sentences. The calculation formula of corpus vocabulary is as follows:

(2) $$\begin{array}{c} W=\left\{W1,W2,\ldots ,Wn\right\}. \end{array}$$

In the above formula, *W* stands for glossary. If *V* is used to represent word vector, there are

(3) $$\begin{array}{c} V_{s}^{i}=\left\{0,0,0,0,1,\ldots ,0\ldots ,0\right\}xu. \end{array}$$

In combination with the curriculum and characteristics of academic foreign language teaching for postgraduates, the WeChat official account of “Yutong future” is designed and established, which contains five modules: management notice, flipped classroom, listening and reading training, learning metastrategy, and emotional interest. Discipline teachers, lecturers, foreign teachers, and graduate assistants are, respectively, responsible for building a bridge between teachers, students, and learning communities. Flipped learning content is directly pushed to learners' WeChat to realize mobile ubiquitous learning. However, the logical fracture and irrelevance between face-to-face course content and online learning content will affect the effect of students' learning with online content [19]. *X* stands for matrix, and *X*_*ij*_ stands for the number of times that words *i* and *j* appear in a window together. Suppose there is a corpus:

(4) $$\begin{array}{c} C=\left\{\text{Tom},\text{I},\text{love},\text{you},\text{and},\text{you},\text{too}\right\}. \end{array}$$

Each time you slide, there is a window content. If the neural network model is not used, but the word vector is constructed based on the ratio characteristic, the relevant formula is as follows:

(5) $$\begin{array}{c} {\text{ratio}}_{ijk}=\frac{P_{ik}}{P_{jk}}=\frac{\exp\left(V_{i}^{T}V_{ik}\right)}{\exp\left(V_{j}^{T}V_{jk}\right)}. \end{array}$$

*P* is the probability that the word *k* appears in the context of the word*i, V* represents the vector representation of the current words*i*, *j*, and *k*, *X*_*i*_represents the number of times the word *i*appears, and *X*_*ij*_ represents the number of times the word *k* appears in the context of *i*. There is also the following formula:

(6) $$\begin{array}{c} P_{ik}=\frac{X_{ik}}{X_{i}},\\ X_{i}=\sum_{j=1}^{N}X_{ij}. \end{array}$$

Therefore, online learning content and classroom face-to-face teaching content can be logically connected or expanded to achieve better learning results. The front-end microclass in the flipped classroom module includes learning instructions, learning support, and a series of related resources. The post-micro-class includes three types: live video of the class, detailed explanation and expansion of key classroom knowledge, and presentation and scene reproduction of difficult content in class. Teachers push prepositioned and postpositioned WeChat courses on the WeChat platform according to the time node (Figure 7), which complement the classroom face-to-face teaching content and jointly promote the learning process.

When the interaction between teachers and students has content, motivation, and expanding ways, it also needs to inject emotion. At present, there are some phenomena in the emotional interaction between teachers and students in colleges and universities, such as “mechanical repetition, loneliness and strangeness, and separation and alienation,” so it is necessary to strengthen the construction. The emotional interaction module in the platform is mainly in charge of teaching assistants, which aims to connect academic groups/subject teachers, Chinese teachers, foreign teachers, teaching assistants (successful learners), and graduate English learners. The main content of the module is the mental journey, capricious perception, and emotional life on various academic roads, aiming to establish the social and emotional connection of teachers' and students' lives and give students more psychological support and identity construction and mutual consistency in social groups [20].

### 3.4. Social and Physical Environment

At the department level, the ecological construction of three centers, writing center, extracurricular practice center, and multimedia learning center, also provides a material environment for graduate students' academic English learning. The writing center is committed to continuing the academic writing teaching in the classroom, providing targeted writing skills and knowledge reference, and providing immediate writing feedback so as to enhance students' learning autonomy. The writing center has also become a teaching and research center for writing teachers. The extracurricular practice center provides various situational learning activities and internship opportunities, such as the “simulated international conference performance” in the school and the interschool international academic seminar for college students (sponsored by China Academic English Teaching Society). The multimedia learning center provides convenient and advanced equipment and thoughtful services for teachers' microclass recording, students' simulated performance recording, classroom teaching recording, and so on. The three centers support each other around learners, and each has its own emphasis: the extracurricular practice center provides context for learning objectives, the writing center focuses on the learning process, and the multimedia learning center ensures the reserve and accumulation of knowledge resources.

## 4. Result Analysis

In the past two years, the graduate English teaching group has made progress in scientific research and curriculum construction. A number of foreign experts have conducted regular teaching and discussion for graduate students, and a relatively stable teacher teaching community has been formed. A series of teaching materials and related online courses have been jointly compiled. There have been a number of provincial and university level scientific research projects related to the course, two of which are provincial key projects and have been successfully concluded. The teachers of the graduate teaching department have published a number of relevant academic papers, most of which are high-level publications in related fields.

In order to verify the effect of the design of ecological academic English learning environment for graduate students, we carried out a preliminary exploration based on questionnaires and focus group interviews. In this study, 1049 non-English major first-year postgraduates were selected as subjects to conduct a questionnaire survey on the satisfaction of the curriculum learning environment. In the field of education, provision is usually the integration of technical, educational, and social situations and provisions. Each kind of provision plays a role in different mechanisms. Therefore, the questionnaire survey is divided into five dimensions, which are teaching community, learning community, learning activities, tools and intermediaries, and social and material environment according to the design elements. In order to avoid score convergence, the questionnaire adopts the six-level Likert scale, from 1 to 6, denoting very dissatisfied, dissatisfied, less satisfied, more satisfied, satisfied, and very satisfied, respectively. Among them, very dissatisfied, dissatisfied, and relatively dissatisfied are regarded as dissatisfied in this paper. Satisfactory and very satisfactory are considered satisfactory. A total of 1049 questionnaires were distributed, and 1000 valid questionnaires were collected, accounting for about 89% of the total number of students. Engineering students accounted for 55%, and science, humanities, and art students accounted for 45%. Male and female students accounted for 49% and 51%, respectively. SPSS was used for statistics. After factor analysis and reliability analysis, the reliability coefficient of 32 items in the questionnaire (KMO > 0.5) was *α* = 0.869.

In the satisfaction test of the five elements of the learning environment (as shown in Table 1), postgraduates' overall satisfaction with the learning environment reached 4.7, and their satisfaction with the flipped classroom resources in the tools and intermediary elements was particularly prominent, reaching 4.9, indicating that they generally hold positive opinions on the reform of the learning environment of academic English and believe that the coordination and cooperation of the teacher-student niche has formed a good learning environment and promoted learning. The semistructured group interview in the later stage also confirmed this attitude, which is mainly reflected in the following five aspects.

### 4.1. Enhanced Learning Motivation

Building a teacher community will enable students to obtain more comprehensive “supplies” and increase their learning motivation. The students said: “Academic English requires both academic and language. Different learning resources are brought by multiple teachers. I think it is more interesting and practical than before. At first, I thought it was troublesome to learn a foreign language lesson from so many different teachers, but if I really put myself into it, I can still learn a lot of useful things, know more about the school and be more interested in the major. Professional teachers' lectures give me the motivation to pursue English literature.” Table 2 shows the satisfaction of students' learning motivation.

### 4.2. Cultivate Innovative Thinking and Collaborative Spirit

Building a learning community is suitable for experiential learning and helps to cultivate graduate students' independent research ability and sense of teamwork. The students said “Task-based learning is very good, because in the past, we used to study for the purpose of examination. We studied and reviewed by ourselves, but we forgot what (knowledge) we had. This kind of cooperation, we wrote (Papers) while learning, and the final report and presentation had our own thinking, deep impression, and memories. Our group has a learning bully as the team leader. Usually, she is responsible for organizing us to study together and do it separately” [21].  Table 3 shows the training satisfaction of innovative thinking and collaborative spirit.

### 4.3. Enhance Learning Investment and Learning Efficiency

Learning activities enable students to clarify their learning objectives and enhance their learning investment and learning efficiency. “We participated in the simulated academic conference competition, but we were defeated. It does not matter. We think (ourselves) speak very well and surpass ourselves.” “I have participated in international conferences of this major, but the meetings are quite watery. Everyone reads them and no one asks questions. The host asks one or two questions (and it is over). I think this simulated academic conference is quite like a foreign conference. Everyone is more natural and more capable for the purpose of communication!” “Before my tutor took me to a foreign conference, I just practiced in the foreign language class and became confident!” Table 4 shows the satisfaction of learning engagement and learning effectiveness.

### 4.4. Promote Personalized Learning

In the aspect of tool intermediary, the flipped classroom and other modules expand the learning space, making the knowledge acquisition more personalized and more in line with the thinking characteristics of graduate students. In the interview, the students said: “with clear extracurricular instructions and guidance, the learning motivation is stronger.” “Knowledge points can be seen by yourself after class. You can participate in more discussions and strengthen understanding in class.” “I prefer the intensive lectures provided by the teachers after class. After class and before the exam, I have a better understanding.” “It's very useful. I've always known that I'm poor and I cannot understand it. But after a semester of training, I can really improve.” Table 5 shows personalized learning satisfaction.

### 4.5. Promote Inquiry Learning and Practical Application Ability

In terms of social and material environment, the students said that the external environment construction is basically perfect, but the internal management and quality hope to be improved. For example, “the seminar room in the library is very convenient, and the teaching assistants and project performance training are conducted there, but there are often no vacancies available” and “they hope to have more field experience, real experience, and the opportunity to go to the factory or enterprise for research in the future.”

According to the comprehensive research, postgraduates hold a positive attitude toward the ecological environment of academic foreign languages. Most students can actively adjust and adapt to the inquiry learning in the postgraduates' stage and have more learning input and stronger learning motivation and cooperation awareness. The overall learning efficiency and the ability to obtain environmental supplies have also been effectively improved.  Table 6 shows the degree of satisfaction with the improvement of inquiry learning and practical application ability.

## 5. Conclusion

The construction of “first-class schools” and “first-class disciplines” in colleges and universities means that future scientific and technological talents must integrate into the international academic circle and have the international discourse power in the field of this discipline. From the perspective of educational ecology, the learning environment of academic English courses for postgraduates should be dynamic, connected, symbiotic, and circular. In this way, the endogenous motivation and external support of learners can be connected through the construction of an ecological learning environment so as to help learners actively obtain ecological “supplies” and achieve the learning effect of complementary disciplinary knowledge and language training. The design of ecological environment needs to build a comprehensive system from the aspects of building teachers' teaching community, students' learning community, learning activities, tool intermediary, social/material environment, and so on. At the same time, the construction of the ecological learning environment of academic English course will also promote cross-international, cross-cultural, and cross-disciplinary cooperation and dialogue and strengthen the connection between the academic community and the world academic circle.

## Figures and Tables

**Figure 1:** Proportion of people engaged in academic research in different industries.

**Figure 2:** Teaching resource sharing mode.

**Figure 3:** Proportion of male and female English teachers.

**Figure 4:** General teaching process.

**Figure 5:** Composition of learning effectiveness.

**Figure 6:** Teaching process of the Mu class.

**Figure 7:** Microclass.

**Table 1:** Satisfaction test results of five elements of learning environment.

Project	Mean value	Quantity (person)	Standard deviation
Teaching community	4.6355	1000	0.6353
Learning community	4.8963	1000	0.2635
Learning activities	4.6987	1000	0.8962
Tool mediation	4.9258	1000	0.3647
Social material environment	4.2536	1000	0.9841

**Table 2:** Satisfaction with learning motivation.

Project	Dissatisfied (*n*/%)	Relatively satisfied (*n*/%)	Satisfied (*n*/%)
With the motivation to pursue literature	15 (1.5)	194 (19.4)	791 (79.1)
More interesting than before	20 (2.0)	310 (31.0)	670 (67.0)
More interested in major	18 (1.8)	240 (24.0)	742 (74.2)

**Table 3:** Training satisfaction of innovative thinking and collaborative spirit.

Project	Dissatisfied (*n*/%)	Relatively satisfied (*n*/%)	Satisfied (*n*/%)
Have your own thinking	20 (2.0)	284 (28.4)	696 (69.6)
With a sense of teamwork	35 (3.5)	273 (27.3)	692 (69.2)
Enhance collaboration	17 (1.7)	338 (33.8)	645 (64.5)

**Table 4:** Satisfaction of learning engagement and learning effectiveness.

Project	Dissatisfied (*n*/%)	Relatively satisfied (*n*/%)	Satisfied (*n*/%)
More investment in learning	17 (1.7)	187 (18.7)	796 (79.6)
Beyond oneself	28 (2.8)	342 (34.2)	630 (63.0)
More effective in learning	31 (3.1)	245 (24.5)	724 (72.4)

**Table 5:** Personalized learning satisfaction.

Project	Dissatisfied (*n*/%)	Relatively satisfied (*n*/%)	Satisfied (*n*/%)
Clearer teacher guidance	47 (4.7)	146 (14.6)	807 (80.7)
Enhanced understanding	30 (3.0)	253 (25.3)	717 (71.7)
Strengthen the foundation	26 (2.6)	332 (33.2)	642 (64.2)

**Table 6:** Satisfaction degree of inquiry learning and practical application ability improvement.

Project	Dissatisfied (*n*/%)	Relatively satisfied (*n*/%)	Satisfied (*n*/%)
Learned to explore	28 (2.8)	200 (20.0)	772 (77.2)
Enhanced practical ability	27 (2.7)	321 (32.1)	652 (65.2)
More involvement in learning	62 (6.2)	257 (25.7)	681 (68.1)

## Data Availability

The labeled dataset used to support the findings of this study is available from the corresponding author upon request.

## References

[1] Liu H., Li X. (2020). Learning path combination recommendation based on the learning networks. *Soft Computing*.

[2] Hejtmanek L., Starrett M., Ferrer E., Ekstrom A. D. (2020). How much of what we learn in virtual reality transfers to real-world navigation?. *Multisensory Research*.

[3] Jin W., Xu R., Lim S., Park D. H., Park C., Kim D. (2021). Dynamic inference approach based on rules engine in intelligent edge computing for building environment control. *Sensors*.

[4] Kim T., Lee J. H. (2020). Reinforcement learning-based path generation using sequential pattern reduction and self-directed curriculum learning. *IEEE Access*.

[5] Li X. (2021). An efficient data evacuation strategy using multi-objective reinforcement learning. *Applied Intelligence*.

[6] Zhao L., Hwang W. Y., Shih T. K. (2021). Investigation of the physical learning environment of distance learning under covid-19 and its influence on students’ health and learning satisfaction. *International Journal of Distance Education Technologies*.

[7] Kariapper R., Samsudeen S. N., Fathima S. (2020). Quantifying the impact of online educational system in teaching and learning environment among the teachers and students. *Solid State Technology*.

[8] Al Amri A. Y., Osman M. E., Al Musawi A. S. (2020). The effectiveness of a 3d-virtual reality learning environment (3d-vrle) on the omani eighth grade students’ achievement and motivation towards physics learning. *International Journal of Emerging Technologies in Learning (iJET)*.

[9] Zhao Y., Tian L., Fan Y., Zhang M., Wang X. (2021). Non-enzymatic glucose biofuel cells based on highly porous ptxni1-x nanoalloys. *Journal of Materials Science*.

[10] Sun P., Wang Y., Laws E., Huang B. (2020). Water mass-driven spatial effects and environmental heterogeneity shape microeukaryote biogeography in a subtropical, hydrographically complex ocean system - a case study of ciliates. *Science of the Total Environment*.

[11] Chai-Arayalert S., Puttinaovarat S. (2020). Designing mangrove ecology self-learning application based on a micro-learning approach. *International Journal of Emerging Technologies in Learning (iJET)*.

[12] Mitra A., Panda S. (2020). Factors affecting usage of internet for academic purpose by university students in smart city bhubaneswar: a sem approach. *High Technology Letters*.

[13] Barkana B. D., Patel A. (2020). Analysis of vowel production in Mandarin/Hindi/american- accented English for accent recognition systems. *Applied Acoustics*.

[14] Li G., Liu F., Sharma A. (2021). Research on the natural language recognition method based on cluster analysis using neural network. *Mathematical Problems in Engineering*.

[15] Pradeep Raj M. S., Manimegalai P., Ajay P., Amose J. (2021). Lipid data acquisition for devices treatment of coronary diseases health stuff on the internet of medical things. *Journal of Physics: Conference Series*.

[16] Liu X., Liu J., Chen J., Zhong F., Ma C. (2021). Study on treatment of printing and dyeing waste gas in the atmosphere with Ce-Mn/GF catalyst. *Arabian Journal of Geosciences*.

[17] Huang R., Zhang S., Zhang W., Yang X. (2021). Progress of zinc oxide-based nanocomposites in the textile industry. *IET Collaborative Intelligent Manufacturing*.

[18] Zhang Y., Kou X., Song Z., Fan Y., Usman M., Jagota V. (2021). Research on logistics management layout optimization and real-time application based on nonlinear programming. *Nonlinear Engineering*.

[19] Zhang Q. (2021). Relay vibration protection simulation experimental platform based on signal reconstruction of MATLAB software. *Nonlinear Engineering*.

[20] Kumar R., Sharma A. (2019). Risk-energy aware service level agreement assessment for computing quickest path in computer networks. *International Journal of Reliability and Safety*.

[21] Ramos D. B., Ramos I. M. M., Gasparini I., Teixeira de Oliveira E. H. (2021). A new learning path model for e-learning systems. *International Journal of Distance Education Technologies*.

